The article "Cultural Connotation and Image Dissemination of Ancient Villages under the Environment of Ecological Civilization: A Case Study of Huizhou Ancient Villages" was retracted in 2023. Reasons: signs of a paper mill; suspected computer-generated content; unreliable results or conclusions; lack of ethics approval or compliance.

# Cultural Connotation and Image Dissemination of Ancient Villages under the Environment of Ecological Civilization: A Case Study of Huizhou Ancient Villages

**DOI:** 10.1155/2022/7401144

**Published:** 2022-08-26

**Authors:** Mingming Zhao, Jun Liang, Shanquan Lu

**Affiliations:** College of Art, Huangshan University, Huangshan 245000, China

## Abstract

Ecological civilization refers to the sum of the material production and consumption mode, social organization and management system, values and ethics, and resource development and environmental influence mode between man and nature created in the practice of transforming nature, adapting to nature, conserving nature, and savoring nature. The construction of ecological civilization is an important part of the realization of the new rural construction goal of “production development, well-off life, civilized village customs, clean village appearance, and democratic management.” With the comprehensive promotion of the construction of a new socialist countryside in China, the ancient villages, as the source foundation of Chinese national culture and the real record of historical information, have become an urgent and severe topic for the current village renovation and protection. This article studies the architectural modeling, village layout, space, color application, and other aspects of ancient Huizhou village architecture, appreciates some elements of form aesthetics, and explores its rich content in modern society, cultural background, and economic conditions. At the same time, starting from the architectural characteristics of ancient Huizhou villages, integrate and understand the characteristics of village layout, architectural shape, and space color application in Huizhou traditional ancient village architecture, and analyze the harmonious beauty, overall beauty, nature, and coordination covered in Huizhou traditional ancient village architecture beauty and other beautiful features. To study the architectural shape, village layout, space, and color application in Huizhou's ancient village buildings, appreciate some elements of morphological aesthetics, and explore its rich content contained in modern society, cultural background, and economic conditions. At the same time, starting from the architectural characteristics of Huizhou ancient villages, we can integrate and understand the characteristics of village layout, architectural shape, and spatial color application in Huizhou traditional ancient villages, and analyze the characteristics of harmony, overall beauty, nature, and coordinated beauty covered in the architecture of Huizhou traditional ancient villages. This study is of great practical significance to promote the comprehensive improvement and protection of historical buildings, traditional residential communities, historical features, and surrounding ecological environment in ancient villages, and to realize the unity of ecology and civilization, efficiency and energy saving, healthy and sustainable development of ancient villages.

## 1. Introduction

The formation of each ancient village has its own factors and conditions, such as its geographical features, natural environment, folk customs, cultural atmosphere, etc. It is these conditions and factors that make traditional and natural villages take on colorful forms. There is a lot of historical and cultural information behind these colorful ancient villages [1].

In the traditional Chinese concept, an ancient village is the interweaving and fusion of people's emotions, and a relatively complete, natural, and traditional ancient village is formed under the gathering of these emotions. The villages that we call “ancient villages” refer to villages with a long history [2]. These villages are built by a huge family system. Here we can not only see the entrepreneurial experience of a certain family, and the legends of the ancestors, but also a record of the rise and fall of the family and the legacy of the ancestors [3]. It can be seen from this that the construction of such a village, an “ancient village,” will follow the ancient Kanyu in the site selection, “paying attention to choosing auspicious places to live.” Kanyu science, which is what people call Feng shui science, that is, the phase technique in the traditional five techniques, is a way to choose the right place. In ancient times, people mainly used it in the selection of palaces, village site selection, house layout and cemetery construction activities, in order to choose a favorable place beneficial to the present and even later generations. Therefore, for the village or the whole village, its layout or single building space, building structure, and building layout are mostly based on the basic idea of “harmony between man and nature” [4]. Taking rivers as the blood of villages and mountains as natural barriers to facilitate people's survival, development and reproduction, ancient villages in my country are widely distributed, as shown in Table 1. As can be seen from the figure, there are 6799 traditional ancient villages in China, among which east China has the largest proportion, 29.9%, followed by southwest China, and northeast China is the smallest with only 0.8%.

Huizhou's ancient villages have a unique charm. This is attributable to the fact that the site selection is based on the ancient theory of kanyu, so first of all, we should pay attention to Feng shui in the site selection of the building. Zhao Jishi, a personage in the Qing Dynasty, once said: “The theory of Feng Shui is especially important for Hui people.” At this time, when building houses, the choice of the homestead and the external environment will be considered together. The “Emperor's House Jingfan House Repair Order” states that “the house takes the situation as the body, the spring water as the blood, the soil as the flesh, and the grass and trees as the hair.” The relationship between the interval, the position of the pool well, the height of the house and the roof, etc., pays attention to the role of “Qi” in the house. For example, Hongcun has Dongshan in the east, Shigu Mountain in the west, Leigang Mountain in the north, and Yangzhan River in the south. Under the embrace of mountains and rivers, Feng shui is unique. However, there is a change in the architectural layout. Since ancient villages are basically based on clan blood relationship, residents with the same surname live together, so the eaves between the same surnames are connected together, but there are also scattered in the gathering. For example, Xidi is scattered and distributed through covered bridges and archways, making the entire village undulating and changing [5]. Once again, the shape is simple and appropriate. The architectural decoration of Huizhou style can be described by blue bricks and black tiles, which not only give people aesthetic enjoyment but also has practical functions of fire prevention, anti-theft, and wind resistance [6]. From the existing topics, we can see that the protection and development of ancient Huizhou villages, or the cultural origins of ancient villages' architectural complexes are mostly discussed, and most of the research content is about architecture, mostly focusing on architectural cases or buildings. In terms of elements, the number of documents is increasing, as shown in Figure1. There is less talk about the influence of the beauty of life forms and aesthetic concepts on architecture in ancient Huizhou villages [7]. Therefore, this article studies the architectural shape, village layout, space, color application, and other aspects of the ancient villages in Huizhou, and analyzes the characteristics of harmony beauty, overall beauty, nature, and coordinated beauty covered in the traditional ancient villages in Huizhou. It is of great practical significance to promote the comprehensive renovation and protection of historical buildings, traditional residential communities, historical features, and the surrounding ecological environment in ancient villages.

## 2. Relevant Theoretical Basis

### 2.1. Conceptual Overview of Village, Ancient Village and Huizhou Ancient Village

The word “village” originated from the description in “Records of the Grand Historian: The Chronicles of the Five Emperors” that “a residence forms a gathering in one year, a city in two years, and Chengdu in three years.” Its commentary points out that “gathering” means the earliest village. Due to the development of society, most people started hunting as the main way of life at that time [8]. Agriculture, forestry, animal husbandry, and sideline fishing have become a comfortable way of life, because agriculture has become a relatively stable production, resulting in the evolution of other villages and towns dominated by agriculture. It became the embryonic form of the village, and as a result, differentiation occurred [9].

“Ancient villages” refer to those villages that once existed and have a historical environment, dating back 5 to 600 years, and their history can be traced back to the Ming and Qing dynasties. Today, the form and layout of ancient villages have undergone major changes. Landscape structure has been valued and respected by modern people [10]. With the increasing emphasis on ancient villages in my country, the number of their identifications has also increased, as shown in Figures 1 and 2. As can be seen from the figure, in all cities, the number of ancient villages in the second and third-tier cities is large, while the number of ancient villages in the first-tier cities is small, mainly because the number of ancient villages is affected by urban construction.

Huizhou Ancient Village is located in the southern part of Anhui Province, at the foot of Huangshan Mountain and by the Xin'an River. Ancient Huizhou governs six counties of Huizhou, Shexian, Jixi, Xiuning, Qimen, and Wuyuan (now in Jiangxi Province). During the Ming and Qing Dynasties, Huizhou Prefecture was basically within the scope of one prefecture and six counties [11]. The residents of “Huizhou Ancient Villages” were mainly scattered by the local Shanyue indigenous people in the early days. Since the Eastern Jin, Tang, and Southern Song periods, the prototype of the ancient villages has gradually formed. Huizhou is close to the Xin'an River, in the south of Anhui and at the foot of Mount Huangshan. It covers the six counties of Yi, She, Xiuning, Wuyuan, Qimen, and Jixi. According to the “Geography of Song Shu”: “In the 3 years of Xuanhe, Shezhou was changed to Huizhou.” There have been various opinions on the place names of Huizhou throughout the ages, and they were named more because of their geographical factors or factors similar to the meaning of words. Geographical factors are nothing more than one is due to the mountains and rivers, and the other is due to the name of the place. For example, Yixian County, which is related to mountains, began in the period of Qin Shihuang, and its name is related to Huangshan, a famous mountain in Anhui. Because the rocks and trees of Huangshan are dark and vigorous, people before and after the Qin Dynasty called it Zhanshan, and later Qin Shihuang set it up [11]. To the south, it was named Zhan County. When Sun Wu of the Three Kingdoms arrived, Zhan Yi became Yi, so the ZIran Mountain in the Qin Dynasty became Yishan. There is She County, which is related to the word “Xi”, “Xi”, which was originally the fusion of water flow, and this place is the confluence of today's Xin'an River and Lianjiang River [12]. Therefore, in the Qin Shihuang period, a county was established here, taking Named She County and so on. “Shanshui Theory” is named Huizhou because there are Huixi and Huiling in Jixi County. This name is recorded in Luoyuan's “Xin'an Zhi” in the Southern Song Dynasty. No matter how the history changed in the later period, this traditional saying has been used all the time. For example, Emperor Qianlong said in “Huizhou Fu Zhi”: Gai County contains Huixi and Huiling. In addition, there is a saying in the “Huizhou Fuzhi” recorded: “Or cloud: Hui, beauty is also, so it is named.” This explanation seems a bit far-fetched on the surface, but if we can think differently or consider it from a positive perspective, most people are more willing to interpret the word “Hui” as beautiful. During the Southern Dynasty, Emperor Liang Wu called “Xin'an is a beautiful landscape”., The Southern Song thinker and writer Zhu Xi once inscribed the word “Xin'an is a great river and mountain” [13]. It can be seen that the names of Huizhou are all related to mountains, rocks, and waters or place names. Because of its long history, it looks ancient. The six counties have been stably affiliated to ancient Huizhou, which is rare in history, especially in Chinese history. We can see or mention the word “Huizhou” in many records, but most of them refer to the word “Huizhou” at this time. “Hui culture” reappears, and “Hui culture” is carried on the land of these six counties, reflecting both the material level and the spiritual side, such as the Hui style architecture, Hui cuisine, Huizhou opera, Huizhou dialect we know, New Security, etc [14]. Among them, Huizhou culture refers to the sum of material civilization and spiritual civilization in one prefecture and six counties of ancient Huizhou but is not equivalent to Anhui culture (Anhui culture is composed of four cultural circles: Huizhou culture, Huaihe culture, Wanjiang culture, and Luzhou culture).

### 2.2. Landscape Ecology

In 1939, the German geographer Troel put forward the concept of landscape ecology. As a popular new interdisciplinary subject, the main body is based on the ecological and geographical theory at the landscape level [15]. It is a discipline that takes landscape and ecology as research topics, including the transmission and sharing of material flow, energy flow, information flow, and value flow on the Earth's surface, and ecosystems formed through the interaction and transformation of biotic and abiotic Principles, structure and function, as well as the use of interactive mechanisms between landscapes and dynamic changes in landscape systems, to study the pattern of landscape aesthetics, optimize the discipline structure, and rationally utilize and protect rural landscapes. The planning and design of beautiful rural landscapes will make rational use of landscape ecology to realize a healthy and harmonious relationship between man and nature, solve rural ecological functions and ecological cycles of rural landscapes, improve the living environment of rural landscapes, and create efficient, healthy and beautiful rural living environment with good ecological benefits [16].

### 2.3. Psychology of Popular Behavior

Mass action refers to collective actions that take place according to to form in mass society and is the sum of many individual responses [17]. The psychology of mass behavior is a synthesis of sociology, psychology, and demand theory, including the hierarchical structure of people [18]. It explores people's desires and behaviors for the environment from the perspective of analyzing human visual information. Research in this area can be done by learning the inner aspirations of rural residents. And better research on rural landscape planning and design. The landscape planning and design of “Beautiful Countryside” must be guided by the psychology of public behavior and adhere to the principle of “people-oriented”. Rural landscape planning and design mainly depend on the approval of the public and villagers, whether it respects public communication and humanistic care, and whether it reflects the potential behavior and psychological awareness of users. Therefore, according to the behavior habits and psychological feelings of users, the needs and habits of people in behavior activities are studied, and then the methods and models suitable for “beautiful countryside” landscape design are summarized [19].

### 2.4. Principles of Landscape Aesthetics

Landscape aesthetics is a discipline that studies the relationship between aesthetic activities. Aesthetic activity is to experience the life of the human image of the world as the object of the activity, and it is the spiritual and cultural activity of human beings. As a branch of aesthetics, landscape aesthetics include landscape design, landscape, psychology, folklore, and other related disciplines. The research process of landscape aesthetics is a process from sensibility to rationality, and then from rationality to practice. Therefore, applying the principles of landscape aesthetics to planning and designing rural landscape design is exactly the process of rising from perceptual cognition to rational cognition, and then putting rational thinking into practice. The process of implementation [20]. In the design, through the landscape change to better reflect the landscape's aesthetic function, to follow the general aesthetic principles, to maximize the maintenance, and strengthen or reshape the formal beauty of the landscape. General aesthetic principles mainly include unification, balance, rhythm, proportion, scale, and other aspects.

## 3. Landscape Research of Ancient Villages in Huizhou

### 3.1. Influencing Factors of the Landscape Formation of Ancient Huizhou Villages

The overall landscape of ancient villages is usually determined by the natural geographical environment where ancient villages are located. For Huizhou, this is particularly prominent. When we analyze the environment of ancient Huizhou villages, we can draw two points:

1. Overall landscape pattern Huizhou's overall landscape pattern is typical of the mountainous areas in southern Anhui. It is composed of the Huangshan Mountains in the middle and its branches on the north and south slopes sandwiched by the river system originating from the Zhongshan Mountains, and the large basins and valleys on the south side of the Huangshan Mountains. It is surrounded by mountains and mountains, and the general trend is from northeast to southwest, with an altitude of about 800 to 1,000 meters. The water flow of Huizhou starts from Shitai County, passes through Huangshan City, and then flows through Taiping Lake all the way to the waters of Qingyi River, and some branches flow through Tunxi and finally to Xin'an River. The location of ancient Huizhou villages and the characteristics of each village show a similar phenomenon
2. Specific landscape environment Huizhou's climate is relatively mild, cloudy and foggy, with little sunshine, and the annual sunshine hours are less than 2000 h; The water in Huizhou is affected by the topography, so the flow of water flowing into the surface is not the same, which will lead to different areas centered on it. So most will take root in places where there is plenty of water but not too much. Huizhou has a suitable environment, so culture thrives here.

According to the overall analysis of Huizhou, we will draw four aspects: first, the impact of the economy on the layout of ancient villages; second, the impact of social systems on the planning of ancient villages; third, the impact of Feng shui on ancient villages; The influence of ancient village planning.

1. Huizhou merchant economy: The spread of the Huizhou merchant economy brought fresh cultural blood to the development of Huizhou villages, and also laid a solid material foundation for the development of villages. With the local influence of Huizhou merchants, it will gradually affect the values around them. The economic development of Huizhou merchants has promoted the economic development of Huizhou ancient villages, which has played a great influence on consolidating the relationship between the clan through various behaviors. At the same time, it develops in education; because the economy promotes cultural prosperity, which also has a significant impact on the interior planning of ancient villages.
2. Clan system: Huizhou patriarchal system is a long-term bred in ancient villages, integrating the social management functions of primitive society, slave society, and feudal society. Its content is complex and far-reaching, and it is a powerful spiritual force and broad ideology as shown in Table 2.
3. Cheng-Zhu Neo-Confucianism: Cheng-Zhu Neo-Confucianism is a type of Neo-Confucian school formed in the Song Dynasty, which has a profound influence on later generations and is a branch of the Neo-Confucian school. Cheng-Zhu's Neo-Confucianism has a wide range of influences, including aesthetics, ideology, etc., so what he pursues is a characteristic of integration with nature. A major feature of ancient Huizhou villages is the “Shuikou Garden,” which is a flexible boundary between ancient villages and the outside world. Cheng and Zhu Neo-Confucianism regards “reason” or “heaven reason” as the highest category of philosophy, and believes that reason is everywhere, which is not only the origin of the world but also the highest criterion of social life. In the theory of human nature, the second course advocates “removing human desire, preserving nature,” and deeply explains this view to make it more systematic.
4. Feng shui culture: Feng shui culture is a kind of mysterious art formed by the Chinese civilization after 5000 years of cultural precipitation. It has rich theories and esoteric essence. The whole set of methodology formed is embodied in the emphasis on “wind and water” in the selection of village sites. Traditional Ancient villages take Feng shui theory as the highest purpose of village site selection and succession. Many plans, layouts, and designs in ancient villages are products of Feng Shui culture.

## 4. Research on the Current Situation and Aesthetic Value of Rural Landscape Construction in Anhui Province

### 4.1. Questionnaire Survey on Rural Landscape Construction in Anhui Province

One of the evaluation criteria of a good landscape design is the understanding of the iron law of “people-oriented” (Table3). The service target of Beautiful Village is the majority of villagers, and the design should be based on the principle of being people-oriented, so this survey is carried out based on the public's satisfaction with Beautiful Village. Since the villagers live in the village every day and have the best understanding of the living environment of the village, it is very important to understand the needs and opinions of the villagers.

Regarding the villagers' understanding of the construction of beautiful villages, more than 40% of the villagers have a good understanding of the construction of beautiful villages, about 30% of the villagers think they understand the construction of beautiful villages, and only a few villagers have not heard about the construction of beautiful villages. Possibilities are shown in Figure 3.

Among the closed-type problems in Shishugang Township, Feixi County, the six items with high dissatisfaction are: the integration of rural site selection with the overall landscape and landform environment, the unity of rural architectural style (color, detail, etc.), the rural agricultural production landscape texture, rural agricultural landscape planting structure (three-dimensional planting and other forms), clean and tidy residential courtyard environment, and residential courtyard greening plant configuration (Figure 4). Through the above results, we can find that Anhui province village for beautiful countryside, and for the village landscape environment is not very satisfactory, it also shows that a lot of ancient village landscape design work did not done because we need to carry out further work in this respect, before the work, we also need to understand the aesthetic value of the ancient village in what aspects.

### 4.2. The Modern Significance of the Aesthetic Value of Ancient Huizhou Villages

So far, aesthetics is no longer the embodiment of appearance, but the expression of spirit, a matter of philosophy. Architectural design is also an aesthetic, it also shows the spiritual and philosophical side. In particular, many modern buildings show some aesthetic characteristics of ancient Huizhou villages.

#### 4.2.1. The Modern Meaning of Overall Beauty

The architectural pattern of ancient Huizhou villages is dominated by residential and courtyard styles. The pink walls, wadai, green mountains, and green waters reflect the beauty of simplicity. The setting of patios and the planning of water streets all reflect the overall beauty of the harmony and unity of humanities and natural landscapes. The overall beauty of this Hui style architecture has also been well applied in modern architecture. Such as the fifth park of Shenzhen Vanke, a modern building. The modern architecture of Shenzhen Vanke No. 5 Park Community appears in the form of a symmetrical axis in the overall planning, and is composed of enclosed courtyards. In the layout of the whole community, the quiet and far-reaching streets and alleys can be seen inside each “village,” if you walk among the paths between courtyards of different sizes, can appreciate the artistic conception and humane neighborhood space.

The simplicity and elegance of Huizhou can be seen from the external image of the building. The first is the shape of the wall, which presents a large solid surface, but this does not affect the space inside the house, nor does it affect ventilation and lighting. The second is the Huizhou style in terms of color, which consistently reflects the abandonment of bright colors and the pursuit of simplicity. Although the large area of white walls is too monotonous, it also provides a good background for various plants.

In the details of the environmental design, efforts are made to create a “quiet” atmosphere in the ancient villages of Huizhou. In the pedestrian planning of Vanke No. 5 Park community, various trees and houses are arranged, such as trees and shrubs are planted, there is a kind of refreshing effect in summer, and there are scattered traveler bananas and plantains with Guangdong characteristics. The dots are dotted among the bushes, reflecting a strong tropical style. There are high and solid walls on both sides of the community streets, and bamboo jungles have been implanted at the side of the road and at the corners, making it not too big. The space appears more secluded, this kind of narrow alleys and deep alleys, against the backdrop of high-walled courtyards, look even more distant.

#### 4.2.2. Guided by the Cultural Market, the Government Should Guide the

Under the background of the rapid development of the modern market economy, through the “invisible hand” of the market, guided by the cultural needs of consumers, the characteristic cultural resources in the region are packaged and integrated, so that cultural advantages are gradually transformed into economic advantages. At the same time, in order to avoid the duplication of construction and disorderly competition between ancient villages and other undesirable phenomena, the local government and tourism authorities should also actively do a good job in guiding, rationally plan the layout, and strengthening the infrastructure construction in scenic spots and surrounding areas. . At the same time, some leading cultural enterprises should be given preferential measures in terms of finance, tax, and fee policies. The design that highlights cultural content and focuses on originality excavates cultural resources with rich connotations and presents them with a new image in front of the world. Whether the content is original or not is a key element that must be paid attention to in the process of designing the cultural resources industry chain of ancient Huizhou villages. Cultural products of original nature often occupy the core competitiveness in the cultural industry chain, and are the elements with the highest added value in the chain. Only by fully excavating local characteristic cultural resources and encouraging cultural creativity in the process of development, can the representative content of these resources be creatively highlighted, and original cultural products with independent intellectual property rights can be produced, scaled, and industrialized. The road. Respecting stakeholders and residents is the most important element in ancient villages. Whether the interests of residents are maintained directly affects the development of local cultural resources. Therefore, the interests of local residents should be placed in the design of the complex cultural industry chain of ancient Huizhou villages. In the first place, safeguard the interests of residents. The design of the cultural industry chain should also give full play to the subjective initiative of the residents of ancient villages, so that they can actively participate in the protection and development of ancient villages, and actively participate in the operation and management of relevant scenic spots. The transformation of cultural resources into cultural benefits enables the participating residents to share considerable benefits and greatly arouses their enthusiasm. This, on the other hand, encourages residents to be more actively involved in the development and protection of ancient villages after obtaining the fruits of interest, thus forming a virtuous circle of interactive ecological protection chains, as shown in Figure 5.

## 5. Conclusion

Based on the ecological civilization of ancient village planning and construction of is a long-term practice, the ultimate goal of our regulation and planning is based on its location conditions, natural conditions, etc., combined with the ecological security, ecological circulation, coordinated population, resources, environment, ecological and comprehensive development of society, for the overall ecological sustainable development of the ancient villages, realize the protection and development of ancient villages, and realize the optimization of resource allocation. This article studies the architectural shape, village layout, space, and color application of the ancient villages in Huizhou, and analyzes the characteristics of harmony, overall beauty, nature, and coordinated beauty covered in the traditional ancient villages in Huizhou. This study is of great reference significance to promote the comprehensive improvement and protection of historical buildings, traditional residential communities, historical features, and surrounding ecological environment in ancient villages, and to realize the unity of ecology and civilization, efficiency and energy saving, healthy and sustainable development of ancient villages.

## Figures and Tables

**Figure 1:** Growth ratio of ancient villages.

**Figure 2:** Determination of ancient villages in batches.

**Figure 3:** Statistical analysis results of the importance of environmental landscape enhancement in the construction of beautiful rural areas.

**Figure 4:** Dissatisfied items of the questionnaire in Shishugang Township, Feixi County.

**Figure 5:** Layered diagram of cultural resources industrialization in ancient Huizhou villages.

**Table 1:** Distribution of traditional ancient villages across the country.

Area	Number of traditional Chinese villages	Proportion of traditional Chinese villages (%)
North China	816	12.00
South China	605	8.90
East China	2031	29.90
Central China	1066	15.70
Northeast China	53	0.80
Northwest China	311	4.60
Southwest China	1917	28.20

**Table 2:** Research on ancient village documents.

year	Number of documents
1990	1
1991	1
1995	2
1996	1
1997	5
1998	6
1999	8
2000	11
2001	9
2002	25
2003	26
2004	38
2005	31
2006	44
2007	70
2008	56
2009	60
2010	78
2011	48
2012	60
2013	69
2014	68
2015	57
2016	74
2017	69
2018	85
2019	83

**Table 3:** List of ancestral halls in ancient villages.

Ancient villages	Ancestral hall
Xidi	Chaimu Hall, diji Hall, huigong temple
Hongcun	Xurentang, shangyuan Hall
Pingshan	Qingyu Hall, chengyi Hall, yaotao Hall, pai god Hall, guangyu Hall
Nanping	Kuiguangtang, xuezhitang, dunbentang, guangxutang
Guanlu	Shidetang
Bishan	Dahontang, mingmutang, qitaitang
Fishing pavilion	Zhongqing Hall, ren Hall, ji Shan Hall, ju qing Hall

## Data Availability

The labeled dataset used to support the findings of this study is available from the corresponding author upon request.
